# Surge Capacity of Taipei's Regional Emergency Medical System during COVID-19: A System Dynamics Approach

**DOI:** 10.1155/2024/5524382

**Published:** 2024-03-14

**Authors:** Chih Chang Chen, Su Ying Hung

**Affiliations:** ^1^Department of Marketing Management, Takming University of Science and Technology, Taipei 11451, Taiwan; ^2^Administrative Center, Taipei Hospital, Ministry of Health and Welfare, New Taipei City 24213, Taiwan; ^3^Department of Information Management, National Taipei University of Nursing and Health Sciences, Taipei 112303, Taiwan

## Abstract

**Background:**

The community transmission of COVID-19 has caused the breakdown of the regional emergency medical system (REMS), impacting the rights and care of regional patients with acute and severe conditions. This study proposes a model for the surge capacity of REMS to plan for readiness and preparedness during challenging events that overload capacity.

**Methods:**

The surge capacity of REMS during the COVID-19 pandemic was studied. The data collection included 26 hospitals that received the data. To simulate the dynamics of Taipei's REMS surge capacity, we observed its ability to treat COVID-19 patients with moderate to severe acute respiratory distress syndrome (ARDS). This will involve monitoring the stock of ventilators, physicians, and nurses within the subsystem loops.

**Results:**

Healthcare managers and administrators can use the overload model and hypothetical scenarios to develop new scenarios with different demands on surge capacity. The REMS system capacity model can be used as an aid to guide planning and cross-checking for address Prepare to plan.

**Conclusions:**

We combined data regarding the availability of ventilators, physicians, nurses, specialized beds, and general acute care beds in our simulations. Thus, our simulations, with support from a well-established regional command and management structure, could help REMS achieve the optimal surge capacity.

## 1. Introduction

Globalization, extreme weather, and population increases have increased the damage of major disasters, such as climate change, earthquakes, infectious diseases, terrorist attacks, and chemical explosions, within a region. Examples of such disasters include the Beirut explosion (2020), the West Sulawesi earthquake (2021), and the COVID-19 pandemic (2019–2022). If the emergency and medical systems of a region fail to sustain their operations during a disaster, the harm inflicted upon the region would far exceed the casualties caused by the disaster itself. Therefore, the surge capacity of regional emergency medical systems (REMS) must be studied in depth.

Studies have been conducted to evaluate the COVID-19 surge capacity of REMS. For example, Barasa et al. [1] performed a simulation analysis under the assumption that 2% of Kenya's population contracted COVID-19; the calculated surge capacity and maximum threshold for general acute care (GAC) beds and intensive care unit (ICU) beds in the REMS indicated a considerable shortage of ventilators and ICU beds. Römmele et al. [2] used the Monte Carlo method to simulate and calculate changes in the demand of REMS for GAC and ICU beds during the COVID-19 epidemic. Litton et al. [3] estimated the surge capacity of ICU beds in Australia's emergency medical system by evaluating the availability of required medical equipment, such as ventilators, hemodialysis machines, intravenous infusion pumps, and extracorporeal membrane oxygenation devices, and health-care professionals, such as physicians and nurses. They identified ventilators, physicians, and nurses to be the primary factors influencing the surge capacity of ICU beds in the REMS. Mateen et al. [4] collected data on ICU and high dependency unit beds in the REMS of England. They employed descriptive statistical methods to calculate a safe threshold value of bed occupancy for admitting patients with COVID-19. This threshold may serve as a reference when revising regional COVID-19 policies. McCabe et al. (2021) modeled the capacity for England's REMS using ventilators, physicians, nurses, general acute care (GAC), and specialist beds. They analysis revealed that the stock of critical care nurses and specialist beds was inadequate to meet the hospitalization requirements of severe ARDS patients during the peak of the COVID-19 epidemic. It was necessary to cancel elective surgeries, establish field hospitals, and recruit personnel to leave. Whether it is retired medical staff or new staff, reallocating and increasing resources (such as adding specialist beds) is essential.

Sánchez-Úbeda et al. [6] performed a case study of hospitals in the Community of Madrid to simulate and predict the demand for GAC and ICU beds. Yamamoto et al. [7] utilize physicians, nurses, respiratory therapists, and ventilators to establish a three-tier model for assessing critical care surge capacity during the COVID-19 pandemic in Japan. They believe that Japan's critical care resources are limited. They suggest that the DMAT headquarters can effectively manage hospital beds and hierarchical medical staff to increase critical care capacity. In addition, they propose converting noncritical care beds, physicians, and nurses into critical care resources to respond to the critical care needs of COVID-19 patients. Chuang [8] stated that the emergency surge capacity of REMS cannot be measured using a single factor, such as the number of available beds. Instead, appropriate standards should be established on the basis of the magnitude of emergency events and the characteristics of hospitals.

The surge capacity of REMS is dependent on wide-ranged, nonlinear, and dynamic feedback and delayed disaster response; thus, effectively measuring the changes in surge capacity by using questionnaires is challenging. Faccincani et al. [9] reported that during emergency situations, the dynamic changes in the surge capacity of REMS are influenced by the status and efficiency of hospital resource utilization. Therefore, evaluating the surge capacity of REMS within a complex dynamic disaster response framework is a challenging task.

Therefore, this study was conducted using a linked framework of used resources and available stock in Taipei's REMS. A comprehensive REMS model was constructed considering the interplay between the number of essential resources, such as ventilators, physicians, and nurses, for treating patients affected by disasters [1–3, 5, 7] and the availability of suitable beds. Analyses were performed using secondary data on daily admissions (August and September 2021) from Taipei's REMS and clinical symptom statistics of patients with COVID-19 reported by Wu and McGoogan [10] and the Taiwanese Ministry of Health and Welfare. Simulations were performed using real-world operational data obtained from Taipei's REMS. Four hypothetical scenarios were simulated to analyze the dynamic changes in the maximum capacity of the REMS for admitting and treating patients with COVID-19 during the study period. Through this study, we hope to gain a comprehensive understanding of the dynamic changes in the operational capacity of Taipei's REMS by analyzing the availability of ventilators, physicians, nurses, specialized beds, and GAC beds. The findings were used to validate the applicability of the REMS [11, 12] and ultimately draw relevant conclusions.

We found that the maximum surge capacity of the REMS is attributable to the availability of system resources including ventilators, physicians, and nurses. This finding is consistent with that of Litton et al. [3]; McCabe et al. [5]; and Yamamoto et al. [7], who stated that the number of ventilators, physicians, and nurses influences the surge capacity of REMS. Our study may serve as a reference for developing effective emergency response plans for REMS. The findings also address the limitations of studies on surge capacity that explored only a single factor [1, 2, 4, 6].

## 2. Model Construction and Hypothetical Scenarios

Barbisch and Koenig [13] first proposed that health-care institutions generate surge capacity through resources such as supplies, manpower, hardware facilities, and command management structures. Sheikhbardsiri et al. [14] reported that enhancing resources, such as physicians, nurses, medical equipment, structures, and systems, may increase the surge capacity of REMS. Chuang [8] emphasized the need for establishing appropriate standards according to the magnitude of mass casualty events and the characteristics of hospitals. Various factors such as overload time and load increase/decrease rate should be used as the basis for planning disaster response plans. Despite the aforementioned studies on the surge capacity of REMS, measuring the influences of surge capacity and the dynamic change in this parameter is challenging.

Given that the surge capacity of REMS is dependent on a dynamic process of delayed response, McLean et al. [12] proposed a system dynamics model for REMS and recommended analyzing the model's fitness and practicality by using real-world disaster data. Zhang et al. [15] conducted a comprehensive study on supply chain logistics, process re-engineering, and system dynamics and proposed using the theory of constraints to simplify complex systems, thereby increasing the feasibility and practicality of system dynamics modeling.

Sarimveis et al. [16] indicated that supply chains and system dynamics are highly similar; many system dynamics models have been used in studies on supply chain management. Caneva [11] suggested that system complexity, which includes aspects such as the number of system components, degree of interconnection, and consistency of change, should be considered when constructing system dynamics models for REMS to address key correlations between events in the modeling and simulation process. Eitel [17] highlighted that constructing a system dynamics model and assessing the changes in model capacity for variables such as beds, physicians, nurses, and other resources may facilitate medical decision-making. Therefore, how simulation data generated through simulations performed using system dynamics models for REMS can be used for decision-making regarding cross-regional natural or anthropogenic disasters must be studied in detail.

Chen [18] developed a regional medical system capacity model to analyze the effects of a surge capacity change in an area affected by the Formosa Fun Coast explosion, using data on medical equipment, medications, physicians, and nursing subsystems loop. Although medications can alleviate symptoms and shorten the treatment duration, as well as increase the monthly medical capacity of the REMS, they do not help to increase the daily surge capacity of the REMS. Hasan et al. [19] After conducting a systematic review of relevant literature on hospital surge capacity preparedness in disasters and emergencies, it is evident that personnel (such as physicians and nurses), materials (medical equipment and drugs), space (GAC or specialized beds), and hospital systems (policies and procedures) all have an impact on surge capacity.

Therefore, for this study, we used a linked framework of used and available key medical resources for treatment in Taipei's REMS. The framework considers the interplay between the availability of essential resources such as ventilators, physicians, and nurses [1–3, 5, 7, 18] and the capacity of GAC and specialized beds for inpatients. This approach allowed us to construct a comprehensive dynamic model of the REMS (Figure 1).

We employ system dynamics modeling to develop a capacity supply chain structure for the REMS. We are analyzing the stock changes in the ventilators, physicians, and nurses subsystems. After deducting the resources required for daily routine medical care, we observed dynamic changes in the maximum surge capacity of REMS. The formula that illustrates the quantitative relationship between the stock loop of beds, ventilators, physicians, and nurses in the capacity model of REMS is as follows.

### 2.1. Stock Description of the Regional Medical Emergency System Capability Model

  TSC_*t*_: Total system capacity of the REMS.
  UCS_*t*_: Used capacity of the REMS on day *t*.
  CSC_*t*_: Number of beds available for inpatients with COVID-19 in the REMS on day *t*.

#### 2.1.1. Description of the Stock Ventilators Subsystem Loop

  TORME_*t*_: Total number of medical equipment in REMS.
  RME_*t*_: The required medical equipment in the REMS on day *t*.
  RMCE_*t*_: The number of medical equipment for COVID-19 inpatients in the REMS on day *t*.

#### 2.1.2. Description of the Stock Physicians Subsystem Loop

  TDS_*t*_: Total number of physicians in the REMS.
  CDS_*t*_: Number of physicians quarantined because of COVID-19 in the REMS on day *t*.
  NDS_*t*_: Number of physicians required for treating inpatients in the REMS on day *t*.
  DTP_*t*_: Number of physicians available for treating COVID-19 inpatients in the REMS on day *t*.

#### 2.1.3. Description of the Stock Nurses Subsystem Loop

  TNS_*t*_: Total number of nurses in the REMS.
  CNS_*t*_: Number of nurses quarantined because of COVID-19 in the REMS on *t*-day.
  NNS_*t*_: Number of nurses required for attending inpatients in the REMS on day *t*.
  NTP_*t*_: Number of nurses available for attending COVID-19 inpatients in the REMS on day *t*.

### 2.2. System Loop Relational Formula

(1) $$\begin{array}{c} {\text{TSC}}_{t}={\text{USC}}_{t}+{\text{CSC}}_{t},\\ {\text{TSC}}_{t}\;-\;{\text{USC}}_{t}={\text{CSC}}_{t},\\ {\text{TSC}}_{t}\;–\;\left({\text{USC}}_{t-1}+{\text{TNONI}}_{t}\;-\;{\text{TNOD}}_{t}+{\text{TNOIC}}_{t}-\;{\text{TNODC}}_{t}\right)={\text{CSC}}_{t}, \end{array}$$

  TNONI_*t*_: detail in the number of inpatients in the REMS on day *t*.
  TNOD_*t*_: Number of inpatients discharged from the REMS on day *t*.
  TNOIC_*t*_: Increase in the number of inpatients with COVID-19 on day *t*.
  TNODC_*t*_: Number of inpatients with COVID-19 discharged from the REMS on day *t*.

#### 2.2.1. Ventilators Subsystem Loop Relational Formula

(2) $$\begin{array}{c} {\text{TORME}}_{t}≧{\text{RME}}_{t}+{\text{RMEC}}_{t}\\ ≧\left({\text{RSV}}_{t}+\alpha_{1}\;{\text{ICUS}}_{t}\;\right)+\alpha_{2}{\text{CSC}}_{t}, \end{array}$$

  RSV_*t*_: Number of patients receiving acute or chronic ventilators therapy in the REMS on day *t*.
 
*α*_1_: Proportion of ICU patients using ventilators in the REMS.
 
*α*_2_: Proportion of inpatients with COVID-19 using ventilators in the REMS.
  ICUS_*t*_: Number of ICU patients in the REMS on day *t*.
  CSC_*t*_: Number of inpatients with COVID-19 in the REMS on day *t*.

#### 2.2.2. Physicians Subsystem Loop Relational Formula

(3) $$\begin{array}{c} {\text{TDS}}_{t}\;-\;{\text{CDS}}_{t}\;-\;{\text{NDS}}_{t}={\text{DTP}}_{t},\\ {\text{DTP}}_{t}\;-\;{\text{NDCS}}_{t}={\text{DTPC}}_{t},\\ {\text{TDS}}_{t}\;-\;{\text{CDS}}_{t}\geq {\text{NDS}}_{t}+{\text{NDCS}}_{t},\\ {\text{TDS}}_{t}\;-\;\left({\text{CSC}}_{t}\times \text{PDI}\times \text{BRNC}\right)\geq \left[\left({\text{USC}}_{t}÷{\text{DBR}}_{t}\right)+\left({\text{CSC}}_{t}\times 2÷{\text{DCPR}}_{t}\right)\right], \end{array}$$

  NDCS_*t*_: Number of physicians required for treating patients with COVID-19 in the REMS on day *t*.
  DTPC_*t*_: Number of physicians available for treating inpatients with COVID-19 in the REMS on day *t*.
  PDI: Number of contacts between patients with COVID-19 and physicians.
  BRNC: Basic reproduction number of COVID-19.
  DBR_*t*_: Ratio of physicians to patients in the REMS.
  DCPR_*t*_: Ratio of physicians to patients with COVID-19 in the REMS.

#### 2.2.3. Nurses Subsystem Loop Relational Formula

(4) $$\begin{array}{c} {\text{TNS}}_{t}\;–\;{\text{CNS}}_{t}\;–\;{\text{NNS}}_{t}={\text{NTP}}_{t},\\ {\text{NTP}}_{t}\;–\;{\text{NNCS}}_{t}={\text{NTPC}}_{t},\\ {\text{TNS}}_{t}\;–\;{\text{CNS}}_{t}\geq {\text{NNS}}_{t}+{\text{NNCS}}_{t},\\ T{\text{TNS}}_{t}-\left({\text{CSC}}_{t}\times \text{PNI}\times \text{PNCI}\right)\geq \left({\text{USC}}_{t}\times 3÷{\text{NPR}}_{t}\right)+\left({\text{CSC}}_{t}\times 3÷{\text{NCPR}}_{t}\right),\\ {\text{TNMS}}_{t}=\left({\text{USC}}_{t}\times 3÷{\text{NPR}}_{t}\right)+\left({\text{CSC}}_{t}\times 3÷{\text{NCPR}}_{t}\right)+\left({\text{CSC}}_{t}\times \text{PNI}\times \text{BRNC}\right)\times {\text{YD}}_{y}÷{\text{WD}}_{y}, \end{array}$$

  NNCS_*t*_: Number of nurses required for attending patients with COVID-19 in the REMS on day *t*.
  NTPC_*t*_: Number of nurses available for attending patients with COVID-19 in the REMS on day *t*.
   PNI: Number of contacts between patients with COVID-19 and nurses.
  BRNC: Basic reproduction number of COVID-19.
  NPR_*t*_: Ratio of nurses to patients in the REMS.
  NCPR_*t*_: Ration of nurses to patients with COVID-19 in the REMS.
  TNMS_*t*_: The total number of nurses required in the REMS in the month.
  YD_*y*_: Total number of days in the year.
  WD_*y*_: Total number of workdays in the year.

Wu and McGoogan [10] analyzed the clinical data of 72,314 patients diagnosed with COVID-19 in China. Approximately 5% of the patients exhibited clinical symptoms of Ventilators failure or septic shock, and an additional 10% exhibited symptoms of hypoxemia, requiring oxygen therapy; 15% of the patients were asymptomatic. The remaining 70% of the patients had mild symptoms and did not require hospitalization. These findings corroborate the statistics (from April 20 to May 30, 2020) compiled by Taiwan's Central Epidemic Command Center regarding community infections caused by the UK variant of COVID-19, which amounted to 7,080 confirmed cases. Among them, 1,055 (14.9%) patients had severe pneumonia or acute Ventilators distress syndrome (ARDS).

In Taiwan, the rate of ventilator usage is high among patients with critical illness and unconscious, long-term bedridden patients. By the end of 2018, the total numbers of ICU beds, subacute Ventilators care beds, and chronic Ventilators care beds in Taiwan were 7,115, 888, and 5,572, respectively. These three types of specialized beds that are equipped with ventilators amounted to a total of 13,573 beds, with approximately 20,000 ventilators available. During the outbreak of the COVID-19 pandemic in Taipei's REMS (May 24, 2021), a total of 9,997 ventilators were available for supporting patients with COVID-19 requiring acute care. Among them, 988 ventilators were still available and ready to deploy, which could accommodate at least 9,880 patients with confirmed COVID-19. In total, 988 patients with COVID-19 had severe ARDS and 1,976 had moderate ARDS. GAC beds in all hospitals in Taiwan are equipped with oxygen supply infrastructure. Therefore, in this study, we evaluated the numbers of intensive care and negative pressure isolation beds available in Taipei's REMS for treating patients with severe symptoms and the number of GAC beds available for treating those with moderate symptoms. Then, the findings were compared with the numbers of available physicians and nurses. Our system dynamics model indicated the changes in the maximum surge capacity of REMS formulas (5) and (6).

(5) $$\begin{array}{c} B_{sr}=\text{MIN }\left\{\left(B_{sr1}\right),\left(D_{sr1}\right),\left(N_{sr1}\right)\right\}, \end{array}$$

(6) $$\begin{array}{c} B_{nr}=\text{MIN }\left\{\left(B_{sr2}\right),\left(D_{sr2}\right),\left(N_{sr2}\right)\right\}, \end{array}$$

 
*B*_*s*_: The maximum number of patients with severe ARDS that can be accommodated in the REMS.
 
*B*_*n*_: The maximum number of patients with moderate ARDS that can be accommodated in the REMS.
 
*B*_*sr*1_: Number of specialized beds available in the REMS.
 
*B*_*sr*2_: Number of GAC beds available in the REMS.
 
*D*_*sr*1_: Number of physicians available in the REMS for admitting and treating the maximum number of  patients with COVID-19 and severe ARDS.
 
*D*_*sr*2_: Number of physicians available in the REMS for admitting and treating the maximum number of patients with COVID-19 and moderate ARDS.
 
*N*_*sr*1_: Number of nurses available in the REMS available for admitting and attending the maximum number of patients with COVID-19 and severe ARDS.
 
*N*_*sr*2_: Number of nurses available in the REMS for admitting and attending the maximum number of patients with COVID-19 and moderate ARDS.

## 3. Hypothetical Scenarios and Simulation

Taipei's REMS, which serves a population of 7 million, has 2,433 specialist beds, 189,178 GAC beds, 2,394 physicians, and 29,659 nurses. Can it meet the medical needs of patients with severe and moderate ARDS during nosocomial infection and community transmission of COVID-19?

We developed four hypothetical scenarios for simulations under the system dynamics model of emergency response, according to a report published by the International Council of Nurses on May 7, 2020. The report indicated that health-care workers with COVID-19 accounted for approximately 6% of the total number of patients with COVID-19 worldwide. The following presents questions proposed based on the four hypothetical scenarios.

1. What is the maximum capacity of the regional emergency medical system to treat patients with COVID-19 and severe ARDS during nosocomial infection periods caused by COVID-19?
2. What is the maximum capacity of the regional emergency medical system to treat patients with COVID-19 and severe ARDS during community spread periods?
3. What is the maximum capacity of the regional emergency medical system to treat patients with COVID-19 and moderate ARDS during nosocomial infection periods caused by COVID-19?
4. What is the maximum capacity of the regional emergency medical system to treat patients with COVID-19 and moderate ARDS during community spread periods?

### 3.1. Simulation of a Regional Medical Emergency System Capacity Model

We collected data from 26 hospitals in Taipei's REMS, covering Taipei City, New Taipei City, Keelung City, and Yilan County. Data were collected between August 1, 2020, and September 30, 2020 (total duration, 61 days) and comprised the following information: monthly statistics of the availability of internal medicine physicians, nurses, and different types of bed (Table 1); daily utilization of different types of beds; and standard ratios of physicians and nurses to beds at the health-care institutions (Table 2).

Using the daily data corresponding to occupied hospital beds of each type, proportion of ventilators in use, and ratios of physicians and nurses to patients, we calculated the dynamic changes in the maximum surge capacity of the REMS for the daily admission of patients with COVID-19 and moderate and severe ARDS in the aforementioned hypothetical scenarios (see Figures 2 and 3).

For instance, Taipei's REMS utilized 18,562 hospital beds, 1,857 physicians, and 14,219 nurses on August 1, 2020. Taipei's REMS still has 861 specialist beds, 6,830 GAC beds, 602 physicians, and 5,054 nurses. Assuming that nosocomial infections occur in 27 wards of Taipei's REMS, it could lead to the quarantine of 135 physicians and 675 nurses, rendering them unable to work. It was estimated that 861 hospitalized patients with severe ARDS and 4073 hospitalized patients with moderate ARDS could receive inpatient treatment. Assuming community transmission occurs within Taipei's REMS, 31 physicians and 155 nurses will require isolation treatment and will be unable to work. It is expected that 861 patients with severe ARDS and 4,260 patients with moderate ARDS could receive inpatient treatment.

Simulations performed using the system capacity model revealed that the REMS exhibits a holiday effect in terms of the utilization of GAC beds. During weekends and holidays, a downward trend can be noted in the number of inpatients, which reaches its lowest point on the weekends after reaching a peak. Specifically, during the holiday period around the Mid-Autumn Festival, a significant decline can be seen in the number of inpatients, which, in turn, enhances the capacity of the REMS for treating patients with COVID-19 and moderate ARDS following the holiday period.

However, this holiday effect does not apply to specialized beds. The surge capacity of Taipei's REMS for treating patients with COVID-19 and severe ARDS is primarily dependent on the availability of specialized beds and ventilators. During both the community spread and nosocomial infection periods, the numbers of ventilators, physicians, and nurses available for admitting and treating patients with COVID-19 and severe ARDS remain sufficient, up to the maximum capacity of specialized beds. For admitting and treating patients with COVID-19 and moderate ARDS, the surge capacity depends on the availability of nurses.

Simulations performed using system dynamics models may enhance our understanding of the dynamic changes in the availability of specialized beds, GAC beds, physicians, and nurses. The results of the simulations performed in this study may guide official decision-making regarding the allocation of temporary beds, procurement of ventilators, provision of additional nursing staff support, and between-region transportation of patients.

## 4. Discussion

We employ two levels of surge capacity: the stock of ventilators, physicians, nurses, and specialized beds available to treat severe ARDS patients, and the stock of physicians, nurses, and GAC beds available to treat moderate ARDS patients [5], to understand the dynamic changes in conventional and surge capacity of the REMS. Comprehensively understanding the real-time changes in the stock of ventilators, physicians, nurses, specialized beds, and GAC beds can serve as a valuable reference for REMS and hospital managers when making decisions [9].

We have found that the effectiveness of REMS in treating severe ARDS patients with COVID-19 largely depends on the stock of ventilators, physicians, nurses, and specialized beds [3, 5, 7]. The surge capacity for treating patients with moderate ARDS is limited by the stock of nurses [5]. For example, on August 1, 2020, 135 doctors and 675 nurses were quarantined due to hospital-acquired infections and were unable to go to work. It is expected that 861 patients with severe ARDS and 4073 patients with moderate ARDS will be admitted. This resulted in a reduction in surge capacity for admitting 197 patients with moderate ARDS compared with clarity.

Just as the explosion occurred at Formosa Fun Coast on June 27, 2015, 449 individuals remained hospitalized for treatment, and 255 were admitted to the intensive care unit, causing an overload at Taipei's REMS specialized beds [18]. Director Huang of the National Health Insurance Administration at Taiwan's Ministry of Health and Welfare publicly urged patients with nonemergency serious illnesses at a press conference on July 2, 2015, not to seek the emergency room of a hospital under Taipei REMS. This was done in order to alleviate the burden of routine medical care. As a result of the COVID-19 community outbreak in mainland China in the fourth quarter of 2019, the number of hospitalizations in Taiwan decreased significantly to 220,000 in the first quarter of 2020, marking a 15% decrease compared to the same period in 2019. For example, on August 1, 2020, Taipei's REMS originally utilized 12,087 GAC beds. After reducing the load by 15%, it is estimated that there will be an increase of approximately 1,813 GAC beds, 181 physicians, and 680 nurses. It can treat an additional 257 patients with moderate ARDS. Therefore, the use of GAC beds in Taipei's REMS showed a holiday discharge effect. This effect slightly increased the system's capacity to accommodate the influx of moderate ARDS [5] following the holidays.

This is consistent with Faccicani et al. [9], who argued that the surge capacity of medical institutions during disaster relief depends on the utilization rate of existing resources. Understanding the impact of the stock of physicians and nurses (personnel), medical equipment (materials), specialized and GAC beds (space) on surge capacity can enhance the quality of processing procedures and policies within the system [19], leading to improved surge capacity in the REMS.

## 5. Conclusions

In this study, a system dynamics model was used to comprehensively analyze the dynamic changes in the surge capacity of the REMS for admitting and treating patients with COVID-19 and moderate and severe ARDS who require GAC or specialized beds.

After analyzing the impact of the availability of physicians and nurses (personnel), ventilators (materials), specialized beds, and GAC beds (space) on surge capacity through simulation. It can serve as a reference for REMS and healthcare facility managers when developing appropriate response strategies. For example, when REMS reaches full capacity, patients will be transferred to nearby REMS facilities [7]. Routine nonemergency and critical care will be reduced, retired medical volunteers will be recruited, field beds will be set up [5], and ventilators will be obtained to enhance REMS surge capacity.

Our findings are consistent with those of Litton et al. [3] and Yamamoto et al. [7] in that the numbers of ventilators, physicians, and nurses affect the surge capacity of ICU beds in REMS. We addressed the limitations of studies on surge capacity that explored only a single factor [1, 2, 4, 6].

Unlike these studies, which conducted simulations for REMS, we combined data regarding the availability of ventilators, physicians, nurses, specialized beds, and GAC beds in our simulations by simulating actual operating data. This allows REMS and healthcare facility managers to precisely capture the dynamics of surge capacity within a REMS, empowering them to make well-informed decisions. REMS can improve their surge capabilities with the support of a robust regional command and management structure [13].

This study did not investigate the effect of medication factors [18] that reduce treatment durations on the monthly surge capacity for treating COVID-19 and severe ARDS patients in REMS. It is recommended that future scholars conduct relevant research and discussions.

## Figures and Tables

**Figure 1:** System capacity model of regional medical emergency systems.

**Figure 2:** Surge capacity of Taipei's regional emergency medical system for admitting and treating patients with COVID-19 and severe ARDS.

**Figure 3:** Surge capacity of Taipei's regional emergency medical system for treating patients with COVID-19 and moderate ARDS.

**Table 1:** Availability of physicians, nurses, and various types of hospital beds in Taipei's regional emergency medical system.

Total number of internal medicine physicians	2,394
Acute care beds	12,051
Acute economy beds	154
Acute general psychiatric beds	841
Acute economy psychiatric beds	12
Acute intensive care beds	1,861
Acute burn beds	50
Burn intensive care beds	38
Infant patient beds	327
Beds for infants with moderate to critical illness	44
Negative pressure isolation beds	367
Positive pressure isolation beds	37
General isolation beds	161
Subacute ventilators care beds	199
Chronic ventilators care beds	445
Hospice beds	178
Total number of nurses	29,659
Isolation beds for acute bone marrow transplant	27
Psychiatric outpatient ward	185
Nuclear medicine beds	13
Acute copayment beds (single)	1,857
Acute copayment beds (double)	4,528
Single psychiatric beds (copayment required)	40
Hospice beds (copayment fee required)	85
Chronic care patient beds	146
Chronic care copayment beds (single)	35
Chronic care copayment beds (double)	56
ER observation beds	858
Hemodialysis beds	1,575
Infant cribs	419
Surgical recovery beds	385

**Table 2:** Standard ratios of physicians and nurses to beds in regional emergency medical system institutions.

Bed category		Physician/patient ratio

General beds	Acute care beds	1 : 10
Specialized and other beds		1 : 10
Chronic care beds (*n* < 50)		2 (with 1 physician being a specialist physician)

Bed category		Nurse/patient ratio

General beds	General acute care beds	1 : 8∼1 : 15
	General acute psychiatric care beds	1 : 3

Specialized beds	Intensive care beds	1 : 2
	Burn intensive care beds	1 : 2
	Burn beds	1 : 2
	Infant patient beds	1 : 3
	Beds for infants with moderate to critical illness	1 : 2
	Negative pressure isolation beds	1 : 2
	Positive pressure isolation beds	1 : 12
	Regular isolation beds	1 : 12
	Subacute ventilators care beds	1 : 2
	Chronic ventilators care beds	1 : 12
	Hospice beds	1 : 3
	Isolation beds for acute bone marrow transplant	1 : 3
	Nuclear medicine beds	1 : 3

Others	Surgical recovery beds	1 : 3
	Emergency observation beds	1 : 2
	Hemodialysis beds	1 : 2
	Infant beds	1 : 12
	Psychiatric day care beds	1 : 20

## Data Availability

Data are available upon reasonable request.
